# Phytochemical Profile and Antimicrobial Activities of Edible Mushroom *Termitomyces striatus*

**DOI:** 10.1155/2021/3025848

**Published:** 2021-10-19

**Authors:** Concepta N. W. Sitati, Kenneth O. Ogila, Rebecca W. Waihenya, Lucy A. Ochola

**Affiliations:** ^1^Department of Biological Sciences, School of Pure and Applied Sciences, Mount Kenya University, P.O. Box 1869-30200, Kitale, Kenya; ^2^Zoology Department, School of Biological Sciences, Jomo Kenyatta University of Agriculture and Technology, P.O. Box 62000-00200, Nairobi, Kenya; ^3^Institute of Primate Research, P.O. Box 24481-00502, Karen, Nairobi, Kenya

## Abstract

The mushroom *Termitomyces striatus* is an edible mushroom that grows wildly and belongs to the family Lyophyllaceae. Studies in the last few decades have demonstrated that mushrooms and their active components have beneficial effects on a variety of biological systems. Some mushrooms do exhibit antibacterial properties. Qualitative phytochemical profile was done on the mushroom *Termitomyces striatus* to establish the presence of compounds responsible for important biological activities. This study also investigated the effect of *Termitomyces striatus* extracts on certain bacterial strains that included *Escherichia coli* and *Pseudomonas aeruginosa* representing the Gram-negative bacteria and *Bacillus subtilis* and *Staphylococcus aureus* representing Gram-positive bacteria. The fungi were represented by *Candida albicans* and *Saccharomyces cerevisiae*. The mushroom was collected in western Kenya, air-dried, and crushed into powder, followed by extraction using water, methanol, and dichloromethane (DCM) solvents. Antibacterial and antifungal activities were evaluated using the disc-diffusion method. Qualitative phytochemical screening of the aqueous extract revealed the presence of alkaloids, flavonoids, steroids, sterols, saponins, phenols, carbohydrates, and proteins. The three extracts exhibited antibacterial against tested bacterial strains. The DCM extract revealed higher effects among the bacterial strains tested. The three extracts showed antifungal effects against *C. albicans*. However, both methanol and aqueous extracts did not inhibit growth of *S. cerevisiae*. In conclusion, *T. striatus* extracts are a promising source of novel antimicrobial and antifungal agents.

## 1. Introduction

Since ancient times, wild mushrooms have been used as a source of food [1]. Before the introduction of exotic mushrooms, native mushrooms were highly consumed as vegetables in Kenya [2, 3]. Out of the 42 tribes in Kenya, 38 tribes are known to consume native mushrooms [4]. Wild edible mushrooms have been collected and consumed in Uganda during the rainy season and valued as a traditionally nutritious food. Some of these are *Polyporus tenuiculus*, *Termitomyces tyleranus*, *Termitomyces clypeatus*, *Volvariella speciosa*, and *Termitomyces microcarpus* [5]. *Termitomyces* is a genus of mushrooms from the division Basidiomycota, kingdom Fungi, and family Lyophyllaceae. There are about 30 species within this genus.

Mushrooms have a history of medicinal use spanning over a millennia. Studies in the last few decades have demonstrated that mushrooms and their constituting active components have beneficial effects on a variety of biological systems [6, 7]. A study in [8] indicated the presence of alkaloids in the extracts of wild edible termitophilous mushrooms. In this study, 0.077 mg/g of alkaloids was found in *T. mammiformis* followed by *T. microcarpus* (0.056 mg/g), *T. medius* (0.053 mg/g), *T. badius* (0.052 mg/g), and *T. striatus* (0.050 mg/g), while the least was in *T. heimii* (0.046 mg/g). Phytochemical analysis of *Termitomyces microcarpus* revealed the presence of volatile oil, alkaloid, carotenoid, steroid, triterpenoids, fatty acid, emodins, flavonoid, coumarin, anthracene glycoside, anthocyanadine glycoside, tannins, saponins, glycosides, polyurenoid, and polyoses in the ethereal, methanolic, and aqueous extracts [9–11].

It has also been reported that there are antioxidant and antimicrobial potentials of extracts obtained from four wild mushrooms: *Termitomyces clypeatus*, *Termitomyces robustus*, *Lentinus subnudus* and *Lenzites* species collected in Nigeria [12]. In their study [13], the authors observed that the mushrooms *T. clyeaptus* and *L. squarrosulus* possess considerable quantities of bioactive compounds.

*Termitomyces striatus* is a mushroom from the genus of edible mushrooms which are commonly consumed in Africa and Asia among the mushrooms collected from the wild. The *Termitomyces* mushrooms grow as symbionts in the termite molds [14]. This mushroom contains important phytochemical compounds such as alkaloids [8] and flavonoids [15]. They also have phenols, saponins, and steroids that have been recorded as possessing antifungal effects [16, 17]. The various extracts of this mushroom also possess antioxidant and antimicrobial activity [18].

The objective of this study was to determine the qualitative phytochemical composition of aqueous extracts of *T. striatus* and the antimicrobial effects of the aqueous extract and methanolic and DCM extracts of *T. striatus* on various strains of bacteria and fungi.

## 2. Materials and Methods

### 2.1. Collection of *Termitomyces striatus*

The mushroom was collected from western Kenya, washed, air-dried, and then ground into fine powder awaiting extraction. The mushroom was authenticated from the National Museum of Kenya (REF: NMK/BOT of 31 MAR 2017) and coded voucher specimens were kept for future reference in the Botany Department of the National Museum of Kenya in Nairobi.

### 2.2. Aqueous Extraction of Mushroom

Mushroom powder weighing 300 grams was added to 800 ml of distilled water and boiled for twenty minutes in in a conical flask. It was allowed to cool until it reached room temperature; thereafter the supernatant was removed. It was centrifuged at 5400x gravity for 10 minutes after which it was filtered through Whatman® GF/C glass microfiber filter paper; it was frozen at −15°C and then dried in a freeze-drier. The extract was kept desiccated at 4°C after being weighed.

The percentage yield of the extract was determined according to the expression provided by [19]

(1) $$\begin{array}{c} \text{percentage yield }=\frac{\text{weight of the extract}}{\text{weight of the mushroom powder}}. \end{array}$$

### 2.3. Methanol and Dichloromethane Extraction of Mushroom

Each three hundred grams of mushroom powder was soaked in one liter of methanol and dichloromethane separately and left standing for two days. The extracts were then filtered and the filtrate was concentrated by a rotary evaporator separately. The concentrate was then stored in air-tight containers and refrigerated.

### 2.4. Qualitative Phytochemical Screening of Extracts

The methods used to test for the presence of alkaloids, flavonoids, sterols and steroids, saponins, and tannins were as described in [19, 20].

### 2.5. Determination of Alkaloids

The mushroom sample was stirred with 1% hydrochloric acid (HCL) on a steam bath. The solution obtained was filtered and 1 ml of the filtrate was treated with two drops of Mayer's reagent. The two solutions were mixed and made up to 100 ml with distilled water. Turbidity of the extract filtrate on addition of Mayer's reagent was regarded as evidence for the presence of alkaloids in the extract.

### 2.6. Determination of Flavonoids

To 1 ml of the mushroom extract in a test tube, a small piece of magnesium ribbon was added followed by drop-wise addition of concentrated hydrochloric acid. Formation of pink or magenta red colours indicated the presence of flavonoids.

### 2.7. Determination of Sterols and Steroids

One milliliter of the mushroom extract was put into a test tube in which 0.5 ml of sulphuric acid, acetic anhydride, and chloroform in similar amount was added. A red coloration indicates presence of sterols while a green colour indicated the presence of steroids.

### 2.8. Determination of Saponins

One milliliter of the mushroom extract under test was put into a test tube and 50 ml of distilled water was added. The mixture was then shaken vigorously. Foaming which persists on warming was taken as an evidence for the presence of saponins. However, the results went through further test for confirmation, which involved dissolving of one milliliter of the extract in a mixture of carbon tetrachloride and 4 drops of concentrated sulphuric acid. A blue, green, or red colour accompanied by a pink ring confirmed the presence of saponins.

### 2.9. Determination of Tannins

Extract of the mushroom sample was stirred with 10 ml of distilled water and then filtered. To the filtrate, two drops of 5% iron III chloride (FeCl_3_) reagent was added. Blue-black or blue-green coloration was an indication of the presence of tannins.

### 2.10. Determination of Carbohydrates

This was done using Molisch's test. To 2 ml of extract, 2 drops of alcoholic-naphthol solution was added in a test tube. Formation of violet ring at the junction indicated the presence of carbohydrates.

### 2.11. Determination of Proteins

To 2 ml of the extract, a few drops of concentrated nitric acid were added. Formation of yellow colour indicated the presence of proteins.

### 2.12. Evaluation of Antimicrobial Activities of *T. striatus* Extracts on Selected Pathogens

The various extracts of the mushroom *T*. *striatus* were subjected to tests to evaluate their antibacterial and antifungal activities. These were done by use of the disc-diffusion method. The bacterial strains which were selected were *Pseudomonas aeruginosa*, *Escherichia coli*, *Bacillus subtilis*, and *Staphylococcus aureus*, while the fungi selected for the study were *Candida albicans* and *Saccharomyces cerevisiae*. The organisms were obtained from a culture collection maintained in the Microbiology Laboratory at Mount Kenya University. The purity of the bacteria was tested by culturing on nutrient agar and being maintained on nutrient agar slants.

### 2.13. Preparation of Inocula

The stock cultures were kept on slopes of nutrient agar. The cultures which were used for the experiments were made by picking a loopful of cells out of the stock cultures and putting in test tubes that contained Mueller–Hinton broth (MHB) for bacteria. Meanwhile, Sabouraud dextrose broth (SDB) was used for fungi. They were reactivated by culturing them overnight at 37°C. Cultures were diluted with fresh MHB and SDB and compared with McFarland standard to achieve values corresponding to 2 × 10^6^ colony-forming unit for bacteria [21] and 2 × 10^7^ spores/ml for fungal strain [22].

### 2.14. Evaluation of Antibacterial Activity of the Extracts

This was done by use of the disk diffusion method as described in [23]. The selected strains of bacteria used were *Escherichia coli* (ATCC 25922) and *Pseudomonas aeruginosa* (ATCC 27853) representing the Gram-negative bacteria and *Staphylococcus aureus* (ATCC 25923) and *Bacillus subtilis* (ATCC 6633) representing the Gram-positive bacteria.

Sterile filter paper discs (Whatman No.1) with a diameter of 5 mm were soaked with mushroom extracts at the concentrations of 6.25, 12.5, 25, 50, 100, and 200 mg/ml. The disks which were soaked in dimethylsulfoxide represented the negative controls [24]. All the bacteria were incubated at 30°C for 24 hours by inoculation into nutrient broth. Sterilized Petri dishes were inoculated with 0.01 ml of one of the above culture media (10^5^-10^6^ bacteria per ml). Mueller–Hinton agar sterilized in a flask and cooled to 45–50°C was distributed in all the Petri dishes that had been inoculated; this was then swirled to enable the medium to be distributed homogenously. The disks which had been injected with the mushroom extracts were placed on the solid agar medium by pressing gently. Ciprofloxacin 0.2 mg/ml [25] was used as the standard drug for the test bacteria strains. The Petri dishes which were treated were kept at 4°C for 1-2 hours and thereafter they were incubated at 35°C for 18–24 hours. The experiments were done in triplicate. When the set time elapsed, the zones of inhibition which had been formed on the media were measured with a transparent ruler in millimeters.

### 2.15. Test of the Mushroom Extracts for Antifungal Activity

The experiments were done using the protocol described in [26] with few modifications. The culture medium was prepared using Sabouraud dextrose agar. The preparation was done in accordance with the manufacturer's direction. The medium was prepared in the conical flask, boiled, and then sterilized by autoclaving. The sterilized medium was cooled to around 50 and exactly 20 ml was dispensed into sterile Petri dishes and allowed to solidify. Thereafter,*. Candida albicans* (ATCC 90028) and *S. cerevisiae* were aseptically inoculated on Petri dishes which were then incubated at 31°C for 48 hours to give white round colonies against a yellowish background. The well isolated colonies of the fungal strains were scooped by help of a sterile wire loop and suspended in sterilized 0.9% sodium chloride solution (normal saline). The turbidity of the inoculum was compared to McFarland solution. The microbial suspension (1 ml) in normal saline was added to 74 ml of sterile medium, kept at 45°C to give concentration of 2 × 10^7^ cells/ml. Sterilized Petri dishes (9 cm diameter) were inoculated with 1 ml of fungal strains. Into the Petri dish containing 1 ml of the fungal strains, 15 ml of the sterile SDA media was added and swirled to mix the fungal strain and the media homogenously. Disks impregnated with extracts at concentrations of 6.25, 12.5, 25, 50, 100, and 200 mg/ml were laid on the solid Sabouraud dextrose agar medium with the help of a sterile pair of forceps and gently pressed. The treated Petri dishes were placed at 4°C for 1-2 hours and then incubated for 48 hr at 37°C. Nystatin 0.2 mg/ml was used as the reference drug [27]. At the end of the period, the inhibition zones formed on the media were measured with a transparent ruler in millimeters.

### 2.16. Statistical Data Analysis

Raw data was recorded in a data book, entered in Microsoft Excel spreadsheet, and then exported to STATA statistical software version 14.2 for analysis. Descriptive statistics were expressed as mean ± standard deviation. One-way analysis of variance was used to determine the statistical difference among different treatment groups followed by Bonferroni post hoc test for comparison of means of different treatment groups. The level of significance was set at 95% (*p* ≤ 0.05).

## 3. Results

### 3.1. Yields of *T. striatus* Extracted

The aqueous extract of *T. striatus* recorded higher yields of 16.0%, followed by dichloromethane with a yield of 6.5%, while methanol extract had the least yield of 3.4% (Figure 1).

### 3.2. Qualitative Phytochemical Analysis

The qualitative screening of aqueous extract of *T. striatus* showed that the following compounds were present: alkaloids, flavonoids, sterols and steroids, saponins, phenols, carbohydrates, and proteins. However, the tannins were absent (Table 1).

### 3.3. Antibacterial Activities of Dichloromethane, Methanol, and Aqueous Extracts on Selected Bacterial Strains

The DCM extract revealed antibacterial activity against *P. aeruginosa*, *E. coli*, *B. subtilis*, and *S. aureus* at concentrations of 6.25, 12.5, 25, 50, 100, and 200 mg/ml. This was indicated by various zones of inhibition of greater than 5 mm in diameter after impregnation of paper discs. The negative control (DMSO) recorded no antimicrobial effect against all bacteria strains tested (Table 2). The antibacterial activity of the reference drug, ciprofloxacin, was significantly higher compared to that of DCM extract at all concentrations tested against all the bacterial strains used (Table 2; *p* < 0.05).

The antibacterial activity of DCM extract against *P. aeruginosa* was significantly higher at the concentrations of 12.5, 25, 50, 100, and 200 mg/ml than that of 6.25 mg/ml (Table 2; *p* < 0.05). Similarly, the antibacterial activity of the DCM extract at concentrations of 50, 100, and 200 mg/ml was significantly higher than that of 6.25 mg/ml against *E. coli* and *S. aureus* (Table 2; *p* < 0.05). However, the antibacterial effect of DCM extract at all concentrations tested showed no significance on *B. subtilis* (Table 2; *p* > 0.05).

The methanolic extract revealed antibacterial activities at different concentrations tested against *P. aeruginosa*, *E. coli*, *B. subtilis*, and *S. aureus*. However, the MeOH extract never revealed antibacterial activity against *E. coli* at the concentration of 6.25 mg/ml (Table 3). The antibacterial effect of the ciprofloxacin was significantly higher compared to that of MeOH extract at all the concentrations tested against *P. aeruginosa*, *E. coli*, *B. subtilis*, and *S. aureus* (Table 3; *p* < 0.05). The negative exhibited no antimicrobial activity on all bacteria strains tested (Table 3).

The zones of inhibition of MeOH extract at the concentration of 200 ml/ml were statistically higher than those of 6.25, 12.5, 25, and 100 mg/ml against *P. aeruginosa* (Table 3; *p* < 0.05). Similarly, the antibacterial effect of the MeOH extract at the concentrations of 100 and 200 mg/ml was statistically higher than those of 6.25 and 12.5 mg/ml against *E. coli* (Table 3; *p* < 0.05). However, the zones of inhibition at all concentrations tested were not significantly different against *B. subtilis* and *S. aureus* (Table 3; *p* > 0.05). Further, the effect of the negative control was comparable to the effect of methanol extract at all tested concentration against *S. aureus* (Table 3; *p* > 0.05).

Also, the aqueous extract at higher concentrations revealed antibacterial activity against *P. aeruginosa*, *E. coli*, and *S. aureus*. However, the aqueous extract demonstrated antibacterial effect at all concentrations tested against *B. subtilis* (Table 4). The concentrations of aqueous extract that never showed the antibacterial effect had zones with a diameter of 5 mm (Table 4). The zones of inhibition of the reference drug, ciprofloxacin, were significantly higher compared to those of aqueous extract at all the tested concentrations against *P. aeruginosa*, *E. coli*, *B. subtilis*, and *S. aureus* (Table 4; *p* < 0.05).

The antibacterial effect of the aqueous extract at the concentrations of 50, 100, and 200 mg/ml was not significantly different against *P. aeruginosa* (Table 4; *p* > 0.05). However, the aqueous extract at concentrations of 6.25, 12.5, and 25 mg/ml never showed antibacterial effect and was comparable to the negative control (Table 4; *p* > 0.05).

The zones of inhibition of aqueous extract at the concentrations of 100 and 200 mg/ml were significantly higher than those of 25 and 25 mg/ml against *E. coli* (Table 4; *p* < 0.05). However, the aqueous extract at the concentrations of 6.25 and 12.5 mg/ml never showed the antibacterial effect against *E. coli* (Table 4). The effect of aqueous extract at the concentrations of 6.25, 12.5, and 25 mg/ml was not significant different against *E. coli* and was comparable to that of the negative control (Table 4; *p* > 0.05).

The antibacterial activity of aqueous extract at all concentrations tested was insignificant against *B. subtilis* (Table 4; *p* > 0.05). Besides, the zones of inhibition of aqueous extract at the concentrations of 25, 50, 100, and 200 mg/ml were not statistically different against *S. aureus*. However, the aqueous extract at the concentrations of 6.25 and 12.5 mg/ml never revealed antibacterial activity against *S. aureus* (Table 4). The effect of aqueous extract at all concentrations tested against *S. aureus* was statistically similar to that of the negative control (Table 4; *p* > 0.05).

### 3.4. Antifungal Activities of Dichloromethane, Methanol, and Aqueous Extracts on *C. albicans* and *S. cerevisiae*

The DCM extract demonstrated antifungal activity against *C. albicans* and *S. cerevisiae* at the concentrations of 6.25, 12.5, 25, 50, 100, and 200 mg/ml. Different zones of inhibition of greater than 5 mm were observed after *C. albicans* and *S. cerevisiae* were treated with DCM extract (Figures 2 and 3). The negative control never revealed antifungal activity (Figures 2 and 3).

The antifungal activity of DCM extract at the concentrations of 100 and 200 mg/ml was statistically higher than that of 6.25, 12.5, and 25 mg/ml against *C. albicans* (Figure 2; *p* < 0.05). The effect of DCM extract at the concentrations of 6.25, 12.5, and 25 mg/ml against *C. albicans* was comparable to negative control (Figure 2; *p* > 0.05). The antifungal effect of the reference drug, Nystatin, was significantly higher compared to that of DCM extract at all the concentrations tested against *C. albicans* (Figure 2; *p* < 0.05).

The zones of inhibition of DCM extract at the concentrations of 200 mg/ml were statistically higher than those of 6.25, 12.5, 25, and 50 mg/ml against *S. cerevisiae* (Figure 3; *p* < 0.05). The zone of inhibition of DCM extract at the concentration of 6.25 mg/ml against *S. cerevisiae* was not significantly different from the negative control (Figure 3; *p* > 0.05). The reference drug, Nystatin, never revealed the antifungal effect against *S. cerevisiae* and was comparable to negative control and extract at the concentration of 6.25 mg/ml (Figure 3; *p* > 0.05).

The MeOH extract also reported the antifungal effect against *C. albicans* at all the concentrations tested. However, the MeOH extract revealed no antifungal activity against *S. cerevisiae* at all the concentrations tested (Figures 4 and 5). The antifungal activity of the MeOH extract was not significantly different against *C. albicans* and was comparable to the negative control (Figure 4; *p* > 0.05). However, the antifungal effect of Nystatin was significantly higher compared to that of MeOH extract at all concentrations tested (Figure 4; *p* < 0.05).

Further, the aqueous extract revealed the antifungal effect against *C. albicans* at all the concentrations tested. However, the aqueous extract showed no antifungal activity against *S. cerevisiae* at all the concentrations tested (Figures 6 and 7). The antifungal effect of the aqueous extract was statistically insignificant against *C. albicans* and was comparable to the negative control (Figure 6; *p* > 0.05). However, the antifungal activity of Nystatin was significantly higher compared to that of aqueous extract at all concentrations tested (Figure 6; *p* < 0.05).

## 4. Discussion

The extract of the test mushroom *T. striatus* possessed important phytochemical compounds, alkaloids, flavonoids, steroids, saponins, and phenols which are responsible for various biological activities important in health research [13]. Phytochemical compounds such as saponins, alkaloids, phenolics, steroids, and flavonoids have been reported to possess antibacterial activities [28–30]. Phenolics, flavonoids, steroids, and saponins have also been documented to possess antifungal effects [16, 17]. Also present were carbohydrates and proteins. This was in conformity with studies by Due et al. [31] where they also found that wild edible mushroom *Termitomyces heimii* Natarajan from Côte d'Ivoire mainly contains proteins and carbohydrates. *T. heimii* is a good source of nutrients and it could be utilized in human diet to alleviate undernourishment caused by protein deficiency. These findings concur with the study in [9] and those in [11] whose authors found out that a sample of *Termitomyces microcarpus* when screened revealed the presence of alkaloids, steroids, flavonoids, saponins, and other compounds in the ethereal, methanolic, and aqueous extracts. The results also agreed with a study in [8] which indicated the presence of alkaloids in the extracts of wild edible termitophilous mushrooms. Besides, in their study, Adejumo et al. [15] found out that the *Termitomyces* mushrooms also contain flavonoids.

In the current study, dichloromethane extract showed antimicrobial activity against all test microorganisms (*P. aeruginosa E. coli*, *B. subtilis*, and *S. aureus*) at all concentrations. DCM demonstrates broad spectrum antibacterial activity by affecting both Gram-positive and Gram-negative bacteria. It was also observed that DCM affects both fungi used in the test that is *C. albicans* and *S. cerevisiae.*

The methanolic extract exhibited antibacterial activities at different concentrations tested against *P. aeruginosa*, *E. coli*, *B. subtilis*, and *S. aureus*. However, there was no antibacterial activity against *E. coli* at the concentration of 6.25 mg/ml. The methanolic extract showed antifungal activity effect against *C. albicans* but not *S. cerevisiae.*

Furthermore the aqueous extract demonstrated antibacterial activity against all the bacterial isolates tested. However, there was higher activity in *E. coli* and *B. subtilis*. This shows that aqueous extract like DCM extract exhibits broad spectrum antibiotic activity. However, aqueous extract shows very weak antibacterial activity against *S. aureus.* This differs from the study in [18] in which they found out that hot water extract of both *Auricularia* and *Termitomyces* mushrooms species showed strong antibacterial activity against *S. aureus*.

Furthermore, in their study using Trametes spp and *Microporus* spp mushrooms, [32]; found out that hot water extracts had the strongest antimicrobial activity against all tested organisms as compared to chloroform and ethanol extracts, which suggested that hot water extraction could be capable of producing several antimicrobial compounds such as flavonoids, tannins, and terpenoids. Like the methanolic extract, the aqueous extract shows antifungal activity against *C. albicans* but not *S. cerev*isiae.

Comparatively, the antibacterial activity of DCM extract was higher (6.25 mg/ml) than that of the other two extracts that is methanol (12.5 mg/ml) and water (25 mg/ml). This means that the DCM has a higher ability of extracting the secondary metabolites responsible for these activities better than the two.

Test of the extracts with the two fungi showed that only the extracts for dichloromethane had higher activity against *C. albicans* and *S. cerevisiae.* The results for antifungal tests in various mushroom extracts concur with the finding of [33], in which the author found out that the various extracts of mushroom *Termitomyces e*xhibited poor activity against various fungal pathogens which he used in the study (*A. flavus, C. albicans,* and *M. racemosus*). The results are also in conformity with observations by [34] in which he found that aqueous extract had little antifungal activity in the plants (*Asparagus setaceus* Kunth and *Caesalpinia volkensii*).

## 5. Conclusion

This study concluded that the dichloromethane, methanol, and aqueous extracts of *Termitomyces striatus* revealed potent antibacterial effect against Gram-negative (*Escherichia coli* and *Pseudomonas aeruginosa*) and Gram-positive (*Bacillus subtilis* and *Staphylococcus aureus*) bacteria. Similarly, the three extracts demonstrated antifungal effect against *C. albicans*. However, the methanol and aqueous extracts never showed antifungal activities against *S. cerev*isiae. The extracts of *T. striatus*, therefore, may be used as antibacterial and antifungal agent.

## Figures and Tables

**Figure 1:** Percentage yields of *T. striatus* extracts.

**Figure 2:** Antifungal activity of DCM extract on *C. albicans*. Bars with the same letter are not significantly different by one-way ANOVA followed by Bonferroni post hoc test (*p* > 0.05).

**Figure 3:** Antifungal activities of DCM extract on *S. cereviceae*. Bars with the same letter are not significantly different by one-way ANOVA followed by Bonferroni post hoc test (*p* > 0.05).

**Figure 4:** Antifungal activity of methanol extract on *C. albicans*. Bars with the same letter are not significantly different by one-way ANOVA followed by Bonferroni post hoc test (*p* > 0.05).

**Figure 5:** Antifungal activities of methanol extract on *S. cereviceae*. Bars with the same letter are not significantly different by one-way ANOVA followed by Bonferroni post hoc test (*p* > 0.05).

**Figure 6:** Antifungal activity of aqueous extract on *C. albicans*. Bars with the same letter are not significantly different by one-way ANOVA followed by Bonferroni post hoc test (*p* > 0.05).

**Figure 7:** Antifungal activities of aqueous extract on *S. cereviceae*. Bars with the same letter are not significantly different by one-way ANOVA followed by Bonferroni post hoc test (*p* > 0.05).

**Table 1:** Qualitative phytochemical analysis of aqueous extract of *T. striatus*.

Substance	Present/absent
Alkaloids	+
Flavonoids	+
Sterols and steroids	+
Saponins	+
Tannins	−
Carbohydrates	+
Proteins	+
Phenols	+

Note: +: present; −: absent.

**Table 2:** Antibacterial activity of DCM extract against *P. aeruginosa*, *E. coli*, *B. subtilis*, and *S. aureus*.

Treatment	Zones of inhibition (mm)			
	*P. aeruginosa*	*E. coli*	*B. subtilis*	*S. aureus*
200 mg/ml	10.67 ± 0.58^b^	7.67 ± 0.58^b^	10.33 ± 1.15^b^	9.33 ± 0.58^b^
100 mg/ml	10.67 ± 0.58^b^	6.50 ± 0.50^bc^	9.33 ± 1.15^b^	9.33 ± 0.58^b^
50 mg/ml	10.33 ± 0.58^b^	6.50 ± 0.50^bc^	9.00 ± 1.00^b^	9.33 ± 0.58^b^
25 mg/ml	9.67 ± 0.58^b^	6.33 ± 0.58^bcd^	9.00 ± 1.00^b^	8.67 ± 0.58^bc^
12.5 mg/ml	9.33 ± 0.58^b^	6.33 ± 0.58^bcd^	8.33 ± 0.58^b^	8.33 ± 0.58^bc^
6.25 mg/ml	7.33 ± 0.58^c^	5.83 ± 0.29^cd^	8.33 ± 0.58^b^	7.67 ± 0.58^c^
Negative control	5.00 ± 0.00^d^	5.00 ± 0.00^d^	5.00 ± 0.00^c^	5.00 ± 0.00^d^
Ciprofloxacin	19.33 ± 0.58^a^	32.67 ± 0.58^a^	20.67 ± 0.58^a^	14.00 ± 0.00^a^

Descriptive statistics expressed as mean ± standard deviation for three replicates. Values with the same letter along the column are not significantly different by one-way ANOVA followed by Bonferroni post hoc test (*p* > 0.05).

**Table 3:** Antibacterial effect of MeOH extract against *P. aeruginosa*, *E. coli*, *B. subtilis*, and *S. aureus*.

Treatment	Zones of inhibition (mm)			
	*P. aeruginosa*	*E. coli*	*B. subtilis*	*S. aureus*
200 mg/ml	8.33 ± 0.58^b^	8.33 ± 0.58^b^	10.66 ± 0.58^b^	5.58 ± 0.38^b^
100 mg/ml	7.33 ± 0.58^bc^	7.33 ± 0.58^b^	10.00 ± 1.00^b^	5.42 ± 0.14^b^
50 mg/ml	6.67 ± 0.58^c^	6.67 ± 0.57^bc^	9.67 ± 0.58^b^	5.42 ± 0.14^b^
25 mg/ml	6.67 ± 0.58^c^	6.33 ± 0.58^bcd^	9.33 ± 0.58^b^	5.33 ± 0.14^b^
12.5 mg/ml	6.33 ± 0.58^cd^	5.83 ± 0.29^cd^	8.67 ± 0.58^b^	5.25 ± 0.00^b^
6.25 mg/ml	6.00 ± 0.00^cd^	5.00 ± 0.00^d^	8.33 ± 0.58^b^	5.25 ± 0.00^b^
Negative control	5.00 ± 0.00^d^	5.00 ± 0.00^cd^	5.00 ± 0.00^c^	5.00 ± 0.00^b^
Ciprofloxacin	19.33 ± 58^a^	31.67 ± 0.58^a^	21.00 ± 1.00^a^	12.33 ± 0.58^a^

Descriptive statistics expressed as mean ± standard deviation for three replicates. Values with the same letter along the column are not significantly different by one-way ANOVA followed by Bonferroni post hoc test (*p* > 0.05).

**Table 4:** Antibacterial effect of aqueous extract against *P. aeruginosa*, *E. coli*, *B. subtilis*, and *S. aureus*.

Treatment	Zones of inhibition (mm)			
	*P. aeruginosa*	*E. coli*	*B. subtilis*	*S. aureus*
200 mg/ml	6.33 ± 0.29^b^	11.67 ± 0.58^b^	7.67 ± 0.58^b^	5.42 ± 0.14^b^
100 mg/ml	6.33 ± 0.29^b^	10.33 ± 0.58^b^	7.67 ± 0.58^b^	5.42 ± 0.14^b^
50 mg/ml	6.17 ± 0.29^b^	8.67 ± 0.58^c^	7.33 ± 0.58^b^	5.33 ± 0.14^b^
25 mg/ml	5.00 ± 0.00^c^	6.33 ± 0.58^d^	7.17 ± 0.29^b^	5.25 ± 0.00^b^
12.5 mg/ml	5.00 ± 0.00^c^	5.00 ± 0.00^d^	7.00 ± 0.00^b^	5.00 ± 0.00^b^
6.25 mg/ml	5.00 ± 0.00^c^	5.00 ± 0.00^d^	7.00 ± 0.00^b^	5.00 ± 0.00^b^
Negative control	5.00 ± 0.00^c^	5.00 ± 0.00^d^	5.00 ± 0.00^c^	5.00 ± 0.00^b^
Ciprofloxacin	19.33 ± 58^a^	32.33 ± 0.58^a^	22.67 ± 1.15^a^	11.67 ± 0.58^a^

Descriptive statistics expressed as mean ± standard deviation for three replicates. Values with the same letter along the column are not significantly different by one-way ANOVA followed by Bonferroni post hoc test (*p* > 0.05).

## Data Availability

The data used to support the findings of this study are available from the corresponding author upon request.
